The article "Computational Intelligence-Based Melanoma Detection and Classification Using Dermoscopic Images" was published in 2022. Journal: Comput Intell Neurosci.

# Computational Intelligence-Based Melanoma Detection and Classification Using Dermoscopic Images

**DOI:** 10.1155/2022/2370190

**Published:** 2022-05-31

**Authors:** Thavavel Vaiyapuri, Prasanalakshmi Balaji, Shridevi. S, Haya Alaskar, Zohra Sbai

**Affiliations:** ^1^College of Computer Engineering and Sciences, Prince Sattam Bin Abdulaziz Univeristy, Al Kharj, Saudi Arabia; ^2^Department of Computer Science, King Khalid University, Abha, Saudi Arabia; ^3^Centre for Advanced Data Science, Vellore Institute of Technology, Chennai, India; ^4^National Engineering School of Tunis, Tunis El Manar University, Tunis, Tunisia

## Abstract

Melanoma is a kind of skin cancer caused by the irregular development of pigment-producing cells. Since melanoma detection efficiency is limited to different factors such as poor contrast among lesions and nearby skin regions, and visual resemblance among melanoma and non-melanoma lesions, intelligent computer-aided diagnosis (CAD) models are essential. Recently, computational intelligence (CI) and deep learning (DL) techniques are utilized for effective decision-making in the biomedical field. In addition, the fast-growing advancements in computer-aided surgeries and recent progress in molecular, cellular, and tissue engineering research have made CI an inevitable part of biomedical applications. In this view, the research work here develops a novel computational intelligence-based melanoma detection and classification technique using dermoscopic images (CIMDC-DIs). The proposed CIMDC-DI model encompasses different subprocesses. Primarily, bilateral filtering with fuzzy k-means (FKM) clustering-based image segmentation is applied as a preprocessing step. Besides, NasNet-based feature extractor with stochastic gradient descent is applied for feature extraction. Finally, the manta ray foraging optimization (MRFO) algorithm with a cascaded neural network (CNN) is exploited for the classification process. To ensure the potential efficiency of the CIMDC-DI technique, we conducted a wide-ranging simulation analysis, and the results reported its effectiveness over the existing recent algorithms with the maximum accuracy of 97.50%.

## 1. Introduction

Computational intelligence (CI) and its wide-ranging applications in biomedical engineering offer oncology, genetic data, genomics, bio-mimetic systems, ontologies construction, protein structure prediction, biomedical data analysis, and biomedical electronics [1]. CI is the study of the design of an intelligent agent, that is a system that can act wisely: they do what they think is applicable for the goal and circumstance; they are flexible to goals and changing environments; they learn from experience, and they make proper selections given finite computation and perceptual limitations. In addition, the rapidly increasing advancement in computer-aided research and surgeries in cellular, tissue, molecular, and engineering makes CI an inevitable part of biomedical applications [2]. The CI paradigm renders more advantages to for enhancing and maintaining the area of biomedical engineering. Skin malignant growth contrasted with other kinds of tumors is a major factor that makes a serious medical illness [3–5]. In earlier years, melanoma was an uncommon malignant growth, but nowadays the total cases of melanoma are increasing dramatically.

To identify skin cancer quickly at the beginning and resolve the abovementioned problems, there is a comprehensive study solution by proposing a computer image analysis algorithm [6]. Most of the algorithmic solution was parametric, which means they needed information to be distributed normally [7]. Since the nature of information could not be controlled, this method will be inadequate to precisely identify the disease. But the nonparametric solution does not depend on the constraints that the information is in standard distribution format. With current advancements in software and hardware techniques, DL is emerging as an effective mechanism for learning features [8]. Feature engineering is a procedure of extracting and determining features by human expertise which is a time-consuming and cumbersome task. The DL method removes the necessity for feature engineering since it is capable of learning and extracting meaningful features automatically from the raw information [9].

DL has transformed various areas, particularly computer vision. In biomedical engineering, DL demonstrates a considerable achievement in the present study. Automatic classification of skin lesions utilizing images is a difficult process because of the fine-grained variation in the appearance of skin lesions. A deep convolution neural network (DCNN) shows potential for highly variable and general tasks through several fine-grained object classes [10]. Outfitted with a deep neural network, the mobile device possibly extends the reach of dermatologists outside of the hospital. The CNN accomplishes performance on par with each testing expert through both tasks, which demonstrates an AI proficiency to classify skin lesions with a level of competencies compared with dermatologists [11].

This study introduces an effective CI-based melanoma detection and classification using the dermoscopic images (CIMDC-DIs) technique. The proposed CIMDC-DI model encompasses bilateral filtering based noise reduction with fuzzy k-means (FKM) clustering based image segmentation as a preprocessing step. Besides, NasNet-based feature extractor with stochastic gradient descent is applied for feature extraction. Finally, realizing the significance of the parameter optimization in enhancing the model performance [12, 13], the manta ray foraging optimization (MRFO) algorithm with cascaded neural network (CNN) is exploited for the classification process. To ensure the better outcomes of the CIMDC-DI technique, a wide-ranging simulation analysis was carried out and the results are assessed under distinct aspects.

## 2. Related Works

Lai et al. [7] presented the technique which combines genomics data, a disease network, and the DL technique for classifying melanoma patients to prognosis, evaluating the influence of genomic features on the classifier, and offering interpretation to impactful features. It combined genomics data with a melanoma network and executed the AE method for identifying subgroups from TCGA melanoma patients. This technique employs community identified from the network to efficiently decrease the dimensionality of genomics data as to patient score profiles. Lafraxo et al. [14] propose a CCN-based deep learning model to automate the classification of benign or malignant skin lesions in dermoscopy images. Furthermore, the performance of the model is improved by utilizing three techniques such as data augmentation, regularization, and dropout to avoid overfitting.

Shorfuzzaman [15] presented an explainable CNN-based stacked ensemble infrastructure for detecting melanoma skin cancer at previous phases. During the stacking ensemble infrastructure, the transfer learning (TL) method was utilized in which several CNN submodels which carry out similar classifier tasks are collected. A novel technique named meta-learner utilizes every submodel forecast and creates the last forecast outcomes. Kim et al. [16] presented a novel unsupervised technique for hair extraction and estimated it on a real-world melanoma data set. During the generative adversarial learning infrastructure, hair feature is considered with coarse-grained label easily utilizing a binary classification. Besides, an essential feature of lesions was well-maintained by minimized L1-norm reconstruction loss dependent upon Laplace noise assumptions.

In [17], a melanoma segmentation method dependent upon DL was presented. In conjunction with post-processed methods, the presented modified U-net network that is extremely effectual from lesions segmentation is established. Hagerty et al. [18] introduced the technique which integrates convention image processing with DL by fusing the feature in the individual approaches. It is offered that two approaches, with distinct error profiles, are synergistic. The convention image processing arm utilizes 3 handcrafted biologically simulated image processing elements and one medicinal data element. In [19], a novel proposal of the DCNN method to classifier skin lesions as malignant and benign on dermoscopic images was presented by creating several connecting blocks for allowing huge feature data to flow directly with the network. All the blocks of the network utilize distinct parameters like the number of kernels, filter size, and stride for extracting low- and high-level feature data in lesions.

## 3. The Proposed Model

This study developed a novel CIMDC-DI approach for melanoma identification and classification using dermoscopic images. The presented CIMDC-DI model involves BF-enabled noise reduction, FKM segmentation, NasNet feature extraction, CNN classifier, and MRFO parameter optimization. The utilization of the MRFO algorithm assists in the effectual choice of parameter values involved in the CNN model.  Figure 1 illustrates the overall block diagram of CIMDC-DI technique.

### 3.1. Bilateral Filtering

At the primary level, the BF technique is used to eradicate the occurrence of noise in dermoscopic images. Dermoscopic images comprise noises like Gaussian, salt pepper noise, and so on [20]. Extracting the noise preserves the data similar to the input data. The BF approach was utilized to denoise this input image. Without utilizing the smoothing edge, the spatial weight averaging was executed by BF. This filtering combines two Gaussian filters to accomplish filtering both in spatial and intensity domain; another one is functioning. In order to weight, both the intensity as well as spatial distances was utilized. The BF output at pixel place *p* is explained as follows:

(1) $$\begin{array}{c} \bar{F}\left(p\right)=\frac{1}{N}\sum_{z\epsilon S\left(p\right)}e\frac{-{\left\|q-p\right\|}^{2}}{2\varepsilon_{e}^{2}}\frac{-{\left|F\left(q\right)-F\left(p\right)\right|}^{2}}{2E_{S}^{2}}F\left(q\right), \end{array}$$

where *S*(*p*) implies the pixel spatial neighbourhood *F*(*p*), *N* denotes the normalized constant, and *ε*_*e*_ and *ε*_*r*_ define the parameters governing weighted from the domains of intensity and spatial begin fall off.

(2) $$\begin{array}{c} e^{\frac{-{\left\|q-p\right\|}^{2}}{2\varepsilon_{e}^{2}}}e^{\;\frac{-{\left|F\left(q\right)-F\left(p\right)\right|}^{2}}{2\varepsilon_{e}^{2}}.} \end{array}$$

The BFs are utilized in texture removal, tone mapping, volumetric denoising, and another application as denoising the images. It creates easy conditions for down-sampling the vital methods and attaining acceleration by expressing under this augmented space by the 2 modest nonlinearity, and the BF was executed as easy linear convolution.

### 3.2. FKM-Based Image Segmentation

In order to identify the lesion regions in the dermoscopic images, the FKM technique has been exploited. The segmentation is employed by an FKM on the extracted set of the melanoma cancer for separating the healthy pixel in the melanoma pixel [21]. The major reason for selecting the FKM over *K*‐means clustering is that *K*‐means clustering is the hard kind of clustering in which one instance belongs to a single cluster; however, in FKM, one instance belongs to one or more clusters; hence, it performs well for overlapped information. The FKM approach separates the image into regions in which *R*_1_(*I*=1,2.3) is associated with the cluster centered *C*_*r*_. FKM has the fuzzy or soft relation among ROI and image and reduces distortion:

(3) $$\begin{array}{c} L=\sum_{j=1}^{k}\sum_{i=1}^{N}b_{ij}^{k}g_{ij}. \end{array}$$

Here, *k* refers the amount of clusters whereas *f* indicates fuzzifier parameter that manipulates the data point and resulting cluster, and *b*_*ij*_ ∈ [0,1] characterizes the relations among the data points and clusters, whereas *g*_*ij*_ characterizes the Euclidean distance amongst data points and clusters.

### 3.3. Feature Extraction

At the time of generating feature vectors, the segmented images are fed into the NasNet model. CNN comprises input and output layers with many hidden convolutional layers. The NASNet model is inspired by Neural Architecture Search (NAS) model [22], which exhibits high flexibility and scalability in terms of computation resources and parameters. It has been trained on the chosen ImageNet database which and is optimized. It comprises a collection of filters, which are then employed to RGB pixel values of the image via sliding window manner. The dot product of filters and input pixels is determined. The feature map is reached in a 2-dimension activation map of the filter.  Figure 2 illustrates the structure of cascaded NN.

It learned the features need to be activated if identified features in the input are attained. Then, the convolutional function is carried out on all feature maps. It enables CNN in learning various feature map weights and biases. Then, max-pooling operation can be utilized for reducing the feature map size. Next to every convolutional layer, subsampling layer is attained which enables to reduction of the size of the convolutional map.

### 3.4. Image Classification

Finally, the MRFO-CNN model receives the features and assigns appropriate class labels to the dermoscopic images. The perceptron connection which is created amongst input as well as output is process of direct relation but in FFNN connection considered among input as well as output is indirect connection [23]. The connection is nonlinear from the shape with activation function under the hidden layer. Once the connection procedure on perceptron and multilayer network was joined, afterward the network with direct connections amongst input as well as output layers was produced, moreover the connection indirectly. The network made in this connection pattern is termed CNN. The formulation developed in CNN approach is demonstrated as follows:

(4) $$\begin{array}{c} y=\sum_{i=1}^{n}f_{i}w_{i}^{i}x_{i}+f^{o}\left(\sum_{j=1}^{k}w_{j}^{o}f_{j}^{h}\left(\sum_{i=1}^{n}w_{ji}^{h}x_{i}\right)\right), \end{array}$$

where *f*^*i*^ refers the activation function in the input to output layers and *ω*_*i*_^*i*^ implies the weight in the input to output layers. Once the bias is extra for input layer and the activation function of each neuron under the hidden layer is *f*^*h*^, then

(5) $$\begin{array}{c} y=\sum_{i=1}^{n}f_{i}w_{i}^{i}x_{i}+f^{o}\left(w^{b}+\sum_{j=1}^{k}w_{j}^{o}f_{j}^{h}\left(w_{j}^{b}+\sum_{i=1}^{n}w_{ji}^{h}x_{i}\right)\right). \end{array}$$

The optimal parameter adjustment of the CNN model is performed by the use of the MRFO algorithm [24]. The MRFO algorithm is stimulated by the fascinating behaviour of the manta rays (MRs). It considers three distinct MR processes like a chain, cyclone, and somersault foraging in providing an efficient optimization approach for identifying solutions to distinct optimization issues. In the MRFO algorithm, the location of the agents can be upgraded at each round via the optimal location of the prey with many planktons, which can be represented as follows:

(6) $$\begin{array}{c} x_{i}^{d}\left(t+1\right)=\left\{\begin{array}{c} \begin{array}{c} x_{i}^{d}\left(t\right)+r\times \left(\left(x_{\text{best}}^{d}\left(t\right)-x^{d}i\left(t\right)\right.\right)\\ \alpha \times x_{\text{best}}^{d}\left(t\right)-x_{i}^{d}\left(t\right)i=1\\ x_{i}d\left(t\right)+r\times \left(\left(x_{i-1}^{d}d\left(t\right)-x_{i}^{d}\left(t\right)\right.\right) \end{array}\\ \alpha \times x_{\text{best}}^{d}\left(t\right)-x_{i}^{d},\left(t\right),i=2,\ldots ,N \end{array}\right., \end{array}$$

where *a* signifies weight coefficient, *r* displays an arbitrary number in [0, 1], *χ*_best_^*d*^(*t*) denotes specific density of plankton, *χ*_*i*_^*d*^(*t*) means location of *i*^th^ and *χ*_*i*−1_^*d*^(*t*) the (*i* − 1)^th^ representatives at iteration *t* in dth dimension, and *α* can be attained using the following equation:

(7) $$\begin{array}{c} \alpha =2r\times \left|\text{log }\left(r\right)\right|1/2. \end{array}$$

The animals create a long bait chain and swim nearer to the bait in case of fixing planktons. The process of storm can be defined in the following:

(8) $$\begin{array}{c} x_{i}^{d}\left(t+1\right)=\left\{\begin{array}{c} x_{\text{best}}^{d}+r\times \left(\left(x_{\text{best}}^{d}\left(t\right)\right.-x_{i}^{d}\left(t\right)\right)\\ +\beta \times \;\left(x_{\text{best}}^{d}\;-x_{i}^{d}\left(t\right)\right)\;,i=1\\ x_{\text{best}}^{d}+r\times \left(\left(x_{i-1}^{d}\right.\left(t\right)-x_{i}^{d}\left(t\right)\right)\\ +\beta \times \left(x_{\text{best}}^{d}\left(t\right)-x_{i}^{d}\right.\;,i=2,\ldots ,N \end{array}\right.,\\ \beta =2\;\exp\left(r_{1}\times \left(\frac{T-t+1}{T}\right)\right)\times \;\sin\left(2\pi r_{i}\right), \end{array}$$

where *T* indicates maximum iteration, *β* displays weight coefficient, and *r*_1_ describes arbitrary numbers among 0 and 1. Bait can be considered as a reference at the time of accomplishing optimal solutions randomly. The storm process can be attained by improving the exploration process in obtaining proper arbitrary location solutions. It can be defined as follows:

(9) $$\begin{array}{c} x_{\text{rand}}^{d}=L^{d}+r\times \left(U^{d}-L^{d}\right),\\ x_{i}^{d}\left(t+1\right)=\left\{\begin{array}{c} x_{\text{rand}}^{d}+r\times \left(\left(x_{\text{rand}}^{d}\left(t\right)\right.-x_{i}^{d}\left(t\right)\right)\\ +\beta \times \;\left(\left.x_{\text{rand}}^{d}\;\left(\text{t}\right)-x_{i}^{d}\left(t\right)\right)\right),i=1\\ x_{\text{rand}}^{d}+r\times \left(\left(x_{i-1}^{d}\left(t\right)\right.-x_{i}^{d}\left(t\right)\right)\\ +\beta \times \left(\left.x_{\text{rand}}^{d}\left(t\right)-x_{i}^{d}\left(t\right)\right)\right)\;,i=2,\ldots ,N \end{array}\right., \end{array}$$

where *χ*_rand_^*d*^ signifies arbitrary location solution and *L*^*d*^ indicates lower and *U*^*d*^ implies higher constraint of the *d*^th^ dimension. The feeding position can be considered as a pivot via somersault foraging. The agents look for somersault and hinge to other locations. Therefore, the positions are considered for attaining optimal positions. Then, it can be represented using the following equation:

(10) $$\begin{array}{c} \chi_{i}^{d}\left(t+1\right)=\chi_{i}^{d}\left(t\right)+S\times \left(r_{2}\times \chi_{\text{best}}^{d}-r_{3}\times \chi_{i}^{d}\left(t\right)\right)\\ i=1,2,\ldots ,N, \end{array}$$

where *S* describes somersault bait and amounts to 2 and *r*_2_ and *r*_3_ display arbitrary numbers. The chaos gets reduced by reducing the distance of the individual planktons. Hence, the somersault forage range reduced with an increase in iterations. In order to choose optimal parameters of the CNN model, the MRFO algorithm has accomplished an objective function, representing a positive integration for implying maximum performance. In this case, the error rate is treated as the fitness function and the solution with minimal error is considered an optimal one. It can be defined as follows:

(11) $$\begin{array}{c} \text{fitness}\left(x_{i}\right)=\text{ClassifierErrorRate}\left(x_{i}\right)\\ =\frac{\text{number of misclassified samples}}{\text{total number of samples}}*100\text{.} \end{array}$$

## 4. Performance Validation

In this section, the experimental validation of the proposed model is performed using three challenging benchmark datasets [25], as shown in Table 1. The results are inspected with 70% of training data and 30% of testing data. A few sample images are demonstrated in Figure 3.

Figure 4 portrays the set of three confusion matrices attained by the CIMDC-DI model on three datasets. On the ISIC2016 dataset, the CIMDC-DI model has recognized 41 images of melanoma and 47 images of benign. Moreover, on the ISIC2017 dataset, the CIMDC-DI algorithm has recognized 55 images of melanoma and 62 images of benign. Furthermore, on the ISIC2017 dataset, the CIMDC-DI approach has recognized 67 images of melanoma and 77 images of benign.

Table 2 provides detailed melanoma classification outcomes of the CIMDC-DI model on the ISIC2016 dataset. The results indicated that the CIMDC-DI model has reported effectual outcomes on both training and testing datasets. For instance, with 70% of the training dataset, the CIMDC-DI model has resulted in average accu_*y*_, prec_*n*_, reca_*l*_, and *F*_score_ of 97.78%, 97.77%, 97.77%, and 97.77%, respectively. Besides, with 30% of the testing dataset, the CIMDC-DI (Table 3) model has accomplished average accu_*y*_, prec_*n*_, reca_*l*_, and *F*_score_ of 94.29%, 94.36%, 94.36%, and 94.29%, respectively.

Table 3 depicts a brief melanoma classification outcome of the CIMDC-DI technique on ISIC 2017 dataset. The results exposed that the CIMDC-DI algorithm has reported effectual outcomes on both training and testing datasets.

For instance, with 70% of the training dataset, the CIMDC-DI methodology has resulted in average accu_*y*_, prec_*n*_, reca_*l*_, and *F*_score_ of 96.79%, 96.85%, 96.84%, and 96.79% correspondingly. Finally, with 30% of the testing dataset, the CIMDC-DI technique has accomplished an average accu_*y*_, prec_*n*_, reca_*l*_, and *F*_score_ of 97.50%, 97.54%, 97.45%, and 97.49%, respectively.

Table 4 offers detailed melanoma classification outcomes of the CIMDC-DI technique on ISIC 2020 dataset. The results demonstrated that the CIMDC-DI method has reported effectual outcomes on both training and testing datasets. For instance, with 70% of training dataset, the CIMDC-DI model has resulted in average accu_*y*_, prec_*n*_, reca_*l*_, and *F*_score_ of 93.14%, 93.16%, 93.18%, and 93.14% correspondingly. Also, with 30% of testing dataset, the CIMDC-DI method has been able average accu_*y*_, prec_*n*_, reca_*l*_, and *F*_score_ of 96%, 96.08%, 95.92%, and 95.98% correspondingly.

A brief precision-recall examination of the CIMDC-DI model on three datasets is portrayed in Figure 5. By observing the figure, it is noticed that the CIMDC-DI model has accomplished maximum precision-recall performance under three datasets.

Figure 6 portrays a clear ROC investigation of the CIMDC-DI model on three datasets. The figure portrays that the CIMDC-DI model has resulted in proficient results with maximum ROC values under distinct class labels.

Table 5 and Figure 7 report the comparative classification outcomes of the CIMDC-DI model with recent models on training phase [26]. The experimental outcomes indicated that the CIMDC-DI technique has outperformed other models in terms of different metrics. On examining the outcome with respect to accu_*y*_,   the CIMDC-DI algorithm has gained higher accu_*y*_ of 96.79% whereas the VGG16, Inception v3, Xception, Inception ResNetV2, and DenseNet121 models have reached lower accu_*y*_ of 90.90%, 88.03%, 91.01%, 93.14%, and 93.30% correspondingly. Besides, on investigating (Table 5) the outcome in terms of prec_*n*_,   the CIMDC-DI technique has gained higher prec_*n*_ of 96.85% whereas the VGG16, Inception v3, Xception, Inception ResNetV2, and DenseNet121 models have reached lower prec_*n*_ of 88.94%, 90.28%, 90.88%, 89.27%, and 92.94%, respectively. Followed by, on investigating the outcome with respect to reca_*l*_, the CIMDC-DI model has gained higher reca_*l*_ of 96.84% whereas the VGG16, Inception v3, Xception, Inception ResNetV2, and DenseNet121 models have reached lower reca_*l*_ of 89.79%, 89.29%, 92.70%, 89.96%, and 91.46% correspondingly.

Table 6 and Figure 8 demonstrate the comparative classification outcomes of the CIMDC-DI technique with recent techniques in testing phase. The experimental outcomes indicated that the CIMDC-DI system has outperformed other models in terms of different metrics. On investigating the outcome with respect to accu_*y*_, the CIMDC-DI methodology has gained higher accu_*y*_ of 97.50% whereas the VGG16, Inception v3, Xception, Inception ResNetV2 (Table 6), and DenseNet121 methodologies have gained minimal accu_*y*_ of 92.75%, 89.61%, 90.49%, 92.80%, and 91.40% correspondingly.

In addition, on examining the outcome in terms of prec_*n*_, the CIMDC-DI approach has gained higher prec_*n*_ of 97.54% whereas the VGG16, Inception v3, Xception, Inception ResNetV2, and DenseNet121 models have achieved decreased prec_*n*_ of 91.25%, 88.50%, 91.16%, 90.53%, and 91% correspondingly. At the same time, on inspecting the outcome with respect to reca_*l*_, the CIMDC-DI model has gained higher reca_*l*_ of 97.45% whereas the VGG16, Inception v3, Xception, Inception ResNetV2, and DenseNet121 models have reached lower reca_*l*_ of 91.58%, 89.24%, 91.36%, 92.99%, and 93.21% correspondingly.

After observing the detailed results and discussion, it is ensured that the CIMDC-DI model has accomplished maximum outcome on melanoma identification and classification using dermoscopic images.

## 5. Conclusion

In this study, a novel CIMDC-DI algorithm was developed for melanoma identification and classification using dermoscopic images. The presented CIMDC-DI model involves BF-enabled noise reduction, FKM segmentation, NasNet feature extraction, CNN classifier, and MRFO parameter optimization. The utilization of the MRFO algorithm assists in the effectual choice of parameter values involved in the CNN model. To ensure the better outcomes of the CIMDC-DI technique, a wide-ranging simulation analysis was implemented and the results are assessed under distinct aspects. A wide-ranging simulation analysis was executed, and the results reported the betterment over the recent methods with the maximum accuracy of 97.50%. Thus, the CIMDC-DI model can be exploited as a proficient tool for real-time melanoma classification. In the future, the CIMDC-DI model can be extended to the incorporation of DL-assisted segmentation approaches. Besides, a fusion-based ensemble classifier model can be developed for melanoma classification.

## Figures and Tables

**Figure 1:** Overall block diagram of CIMDC-DI technique.

**Figure 2:** Structure of cascaded neural network.

**Figure 3:** Sample images.

**Figure 4:** Confusion matrix of the CIMDC-DI model on three datasets.

**Figure 5:** Precision-recall analysis of CIMDC-DI technique under three datasets.

**Figure 6:** ROC analysis of CIMDC-DI technique under three datasets.

**Figure 7:** Comparative analysis of CIMDC-DI technique on training phase.

**Figure 8:** Comparative analysis of the CIMDC-DI technique on testing phase.

**Table 1:** Dataset details.

ISIC 2016 dataset			
Class	Training samples	Testing samples	Total samples
Melanoma	108	42	150
Benign	102	48	150
Total	210	90	300

ISIC 2017 dataset			
Class	Training samples	Testing samples	Total samples
Melanoma	140	60	200
Benign	140	60	200
Total	280	120	400

ISIC 2020 dataset			
Class	Training samples	Testing samples	Total samples
Melanoma	179	71	250
Benign	171	79	250
Total	350	150	500

**Table 2:** Result analysis of CIMDC-DI technique on ISIC 2016 dataset

Class labels	Accuracy	Precision	Recall	*F*-score
Training (70%)				
Melanoma	97.78	97.62	97.62	97.62
Benign	97.78	97.92	97.92	97.92
Average	97.78	97.77	97.77	97.77

Testing (30%)				
Melanoma	94.29	97.06	91.67	94.29
Benign	94.29	91.67	97.06	94.29
Average	94.29	94.36	94.36	94.29

**Table 3:** Result analysis of CIMDC-DI technique on ISIC 2017 dataset.

Class labels	Accuracy	Precision	Recall	*F*-score
Training (70%)				
Melanoma	96.79	99.26	94.41	96.77
Benign	96.79	94.44	99.27	96.80
Average	96.79	96.85	96.84	96.79

Testing (30%)				
Melanoma	97.50	98.21	96.49	97.35
Benign	97.50	96.88	98.41	97.64
Average	97.50	97.54	97.45	97.49

**Table 4:** Result analysis of CIMDC-DI technique on ISIC 2020 dataset.

Class labels	Accuracy	Precision	Recall	*F*-score
Training (70%)				
Melanoma	93.14	94.80	91.62	93.18
Benign	93.14	91.53	94.74	93.10
Average	93.14	93.16	93.18	93.14

Testing (30%)				
Melanoma	96.00	97.10	94.37	95.71
Benign	96.00	95.06	97.47	96.25
Average	96.00	96.08	95.92	95.98

**Table 5:** Comparative analysis of CIMDC-DI technique with recent algorithms on training phase.

Training phase			
Methods	Accuracy	Precision	Recall
VGG16 model	90.90	88.94	89.79
InceptionV3 model	88.03	90.28	89.29
Xception model	91.01	90.88	92.70
Inception ResnetV2 model	93.14	89.27	89.96
DenseNet121 model	93.30	92.94	91.46
CIMDC-DI	96.79	96.85	96.84

**Table 6:** Comparative analysis of CIMDC-DI technique with recent algorithms on testing phase.

Testing phase			
Methods	Accuracy	Precision	Recall
VGG16 model	92.75	91.25	91.58
InceptionV3 model	89.61	88.50	89.24
Xception model	90.49	91.16	91.36
Inception ResnetV2 model	92.80	90.53	92.99
DenseNet121 model	91.40	91.00	93.21
CIMDC-DI	97.50	97.54	97.45

## Data Availability

Data sharing is not applicable to this article as no datasets were generated during the current study.
